The article "Reliability Analysis of a Functional Diagnostic Test for Primary Hyperaldosteronism Based on Data Analysis" was published in 2022. Journal: Comput Intell Neurosci.

# Reliability Analysis of a Functional Diagnostic Test for Primary Hyperaldosteronism Based on Data Analysis

**DOI:** 10.1155/2022/6868941

**Published:** 2022-06-27

**Authors:** Yan Wang, Jun Cai

**Affiliations:** Fuwai Hospital, Chinese Academy of Medical Sciences, Beijing 100037, China

## Abstract

Primary aldosteronism (PA) is one of the most common causes of secondary hypertension, with a prevalence of 12–20% in the hypertensive population. To determine the characteristic function of a fuzzy concept based on the epidemiological data, clinical manifestations, and auxiliary examinations of PA, the essence is to select a suitable domain and determine the affiliation of each element in the domain. The aldosterone/renin ratio was proposed to increase the detection rate of PA, which has the shortcoming of a high underdiagnosis rate when relying only on clinical manifestations. However, there is no unified standard for the diagnostic cut point, and there are differences in testing methods and diagnostic cut point values for different populations, which require different laboratories to establish appropriate cut points according to different regional populations to improve the diagnostic accuracy. In this article, we analyzed the reliability of functional diagnostic tests for PA based on data analysis and compared the sensitivity and specificity of different plasma aldosterone cut points for the diagnosis of PA in the 40 mg kibbutz test. The results showed that when post-saline PAC and post-cato PAC were used to confirm the diagnosis of proaldosterone, respectively, there was a similar subject working area under the curve between SSST and CCT, 0.89 and 0.78, respectively, with no significant difference in the area under the curve between the two (*p*=0.546). Therefore, blood sodium and blood potassium have higher specificity and sensitivity than SUSPUP, but both are lower than ARR, and data analysis can be used as an auxiliary indicator for screening.

## 1. Introduction

PA is a syndrome characterized by hypertension with (or without) hypokalemia due to pathological changes in the adrenal cortex leading to the autocrine secretion of aldosterone, with high plasma aldosterone concentration and low renin as the main biochemical features [1]. PA is characterized by arterial hypertension, spontaneous hypokalemia, hyperkalemia, hyperaldosteronism, and reduced plasma renin activity [2]. With the economic and social development, the prevalence of hypertension is increasing year by year, and epidemiological surveys show that the prevalence of hypertension among adults in China is 31% [3]. It is known that the causes of hypertension include primary and secondary elevated blood pressure, and secondary causes include renal parenchymal, renal vascular, and adrenal and polyarteritis [4]. Substantial renal hypertension is mainly caused by primary or secondary renal lesions, the most common of which would be glomerulonephritis [5]. PA is not uncommon in hypertension, being 15% in severe hypertension (≥180/100 mm Hg) and up to 25% in resistant hypertension [6].

Screening for people at high risk of PA followed by confirmatory tests to clarify the diagnosis and finally typing of PA is an internationally accepted process for the diagnosis of PA [7]. The American College of Endocrinology PA guidelines recommend saline loading test, captopril test (CCT), oral sodium loading test, and fludrocortisone test as the four confirmatory tests for PA [8]. Numerous studies have shown a significantly increased risk of metabolic syndrome and cardiovascular disease in patients with PA compared to patients with essential hypertension [9]. The risk to the organism is much higher than in patients with primary hypertension with the same disease duration and the same degree of blood pressure [10]. Data analysis is mainly a combination of a priori knowledge and available statistical data, using probabilities to predict things [11]. This method is a fundamental approach in statistical modeling and is widely used in medical fields such as oncology, pathology, and high-throughput histology [12]. In this study, we investigated the diagnostic value of data analysis on the reliability of functional diagnostic tests for PA and studied the sensitivity and specificity of different post-dose plasma aldosterone cut points for the diagnosis of PA to provide a more rational basis for clinical diagnosis.

The traditional reliability analysis method is based on the analysis of life data (time to failure) [13]. The statistical analysis of life data determines the type of life distribution of the product and based on that the reliability assessment, prediction, etc. of the product [14]. However, in our clinical work, we found that many patients with essential hypertension had a decrease in blood aldosterone levels <28% from baseline after oral administration of captopril, suggesting that the responsiveness to captopril is lower in national than in Western populations, making it difficult to identify hyporenin-active hypertension from PA in clinical practice based on the guideline-recommended blood aldosterone cut point values [15]. Therefore, as in all other endocrine diseases, functional diagnosis plays an important role in the diagnosis of PA and is the basis for localization and staging.

The innovative points of this study are as follows:

1. This study uses the principles and methods of data analysis to select simple, rapid, and economical tests for the diagnosis of PA and identifies the most common subtypes of aldosteronism in PA.
2. The study explores the optimal aldosterone level for CAPT diagnosis of PA by assessing the degree of suppression of blood aldosterone levels in patients with PA and essential hypertension by CCT and comparing them with normotensive volunteers.
3. The SROC method and data analysis were used to evaluate the diagnostic results of IHA and ELISA, and it was found that the two statistical methods yielded similar conclusions, but the data analysis could yield the mean and confidence interval of sensitivity, specificity, and DOR, respectively, so that the data analysis was more reliable for the functional diagnostic test of PA.

The rest of the article is organized as follows: Section 2 imports the works related to the PA functional diagnostic test and data analysis. Section 3 sorts the PA screening method based on data analysis, and the method of Khyberton inhibition test, so that the readers of this article can have a more comprehensive understanding of the method of PA functional diagnostic test reliability based on data analysis. Section 4 is the core of the thesis, which completes the description of the application analysis of data analysis in PA diagnostic test reliability from two aspects: threshold effect detection analysis and statistical analysis of diagnostic test reliability. Section 5 summarizes the full work.

## 2. Related Works

### 2.1. PA Functional Diagnostic Test

At present, the diagnosis of PA is divided into three parts: first, screening diagnosis followed by the determination of diagnosis and then identification of various subtypes of PA for the selection of treatment. More and more studies have found that in addition to clinical manifestations such as hypertension and hypokalemia, PA can also cause serious damage to the heart, kidney, brain, and blood vessels of patients, and several domestic and international studies have shown that the proportion of cardiovascular disease is higher in patients with PA compared with primary hypertension. In addition, some patients may present with hypokalemia due to the long duration of the disease or after diuretics—weakness, numbness, muscle paralysis, and other discomforts—and target organ complications such as heart, brain, and kidney due to hypertension and high ALD levels.

Rege et al. found significant differences in the expression of genes in the globular and fascicular bands of the rat adrenal gland using gene microarrays, specific expression in the globular band of the rat adrenal gland by immunohistochemistry and other methods, and a close relationship with the expression of enzyme ketone synthase and enzyme ketone secretion [16]. Holler et al. found that some somatic cells in aldosterone adenoma are mutated, resulting in abnormalities in the genes encoding Na-KATPase and Ca2+ATPase that increase adrenal autocrine secretion of aldosterone leading to hypertension [17]. Fuss et al. determined the diagnosis of PA based on clinical presentation, confirmatory tests, and pathological examination [18]. Receiver operating characteristic (ROC) curves for diagnosing PA by ARR in different body positions were constructed and the best cut point for ARR screening of PA was selected according to the Youden's index. Zhang et al. found that during the follow-up of 2000 cases of intractable hypertension, about 13% of patients were confirmed to have PA and were those who could achieve clinically curable hypertension, suggesting that early diagnosis of PA can help to effectively control blood pressure and even end target organ damage caused by hypertension [19]. Freel and Connell considered the value of its application in the diagnosis of primary acid fixation, further assessing its sensitivity and specificity as a screening index by comparing it to the ARR ratio [20].

The probability that a patient with a specific disease has all the clinical manifestations and ancillary findings of this disease is almost small, and the diagnosis can only be made or excluded clinically based on the extent to which the patient's presentation matches all the manifestations. Therefore, the aim of this study was to further investigate the reliability of functional diagnostic tests for PA in a Chinese population by analyzing the data and correcting for relevant confounding factors.

### 2.2. Data Analysis

The clinical manifestations and ancillary findings of a disease are the sum of the results of a large sample of “all patients.” The criteria for diagnosing PA is pathological diagnosis, but it is not required that all hypertensive patients undergo pathological biopsy, so a series of clinical diagnostic strategies are needed. The current diagnostic process of PA mainly includes a screening test, confirmatory test, and localized diagnosis, and this screening test can exclude the influence of other antihypertensive drugs in patients with newly diagnosed hypertension, which has a high diagnostic accuracy and helps to rationalize the use of drugs. However, the results of different studies suggest that the diagnostic efficacy of ADRR in PA screening is highly variable, and it is necessary to analyze the data on the diagnostic efficacy of ADRR in PA to clarify the role of ADRR in prodrug screening.

Gruber et al. used SAS 9.1 for statistical analysis and calculated the results of the study using data analysis, sensitivity, and specificity bivariate model analysis, respectively, and compared the calculated results of the two methods [21]. To assess the overall diagnostic value, Kersten et al. used data analysis for meta-analysis with effect indicators of total sensitivity, total specificity, total positive likelihood ratio, total negative likelihood ratio, diagnostic ratio, and the area under the working characteristic curve of the combined subjects [22]. Studies of Pitt and Byrd exploring the efficacy of ADRR screening for PA were included in the analysis, and two researchers independently extracted and analyzed the study data, which included general patient status and antihypertensive medication use [23]. Funder et al. concluded that reliability analysis through degraded information saved trial time and cost [24]. Reliability analysis based on performance degradation data is one of the solutions to the problem of reliability assessment of highly reliable and long-lived products. Pan et al. used chemiluminescence and data analysis to determine PAC and PRC of 200 hypertensive patients (including 67 patients with PA) in the prone and standing positions for 2 h, and 133 healthy volunteers in the standing position for 2 h, and calculated the ARR of different positions [25].

Therefore, the article explored the value of data analysis in the diagnosis of prodromal by exploring the predictors of prodromal and comparing their laboratory biochemical data in an attempt to construct a mathematical model using data analysis alone or in combination with traditional ARR methods.

## 3. Method of PA Functional Diagnostic Test Reliability Based on Data Analysis

### 3.1. PA Screening Method Based on Data Analysis

Cardiovascular diseases are included in the category of coronary atherosclerotic heart disease (coronary heart disease) and stroke [26]. Among them, coronary heart disease includes two types of stable angina pectoris and myocardial infarction [27]. Diagnostic criteria were used which developed by the Cardiovascular Disease Branch of the Chinese Medical Association [28]. A theoretical domain consisting of elements involving symptoms, laboratory tests, and imaging was selected and determined by reviewing the statistical literature related to PA [29]. The evaluation test diagnosed it as having the disease, and the false positive result put the subject under great mental stress. For the calculation of the above indicators, TPR and FPR were calculated and then logit transformations were applied to TPR and FPR with the following formulas:

(1) $$\begin{array}{c} \log\text{it}\left(\text{TPR}\right)=\ln\left[\frac{\text{TPR}}{\left(1-\text{TPR}\right)}\right], \end{array}$$

(2) $$\begin{array}{c} \log\text{it}\left(\text{FPR}\right)=\ln\left[\frac{\text{FPR}}{\left(1-\text{FPR}\right)}\right]. \end{array}$$

Add two variables D and S, and the expressions are as follows:

(3) $$\begin{array}{c} \text{D}=\log\text{it}\left(\text{TPR}\right)-\log\text{it}\left(\text{FPR}\right), \end{array}$$

(4) $$\begin{array}{c} S=\log\text{it}\left(\text{TPR}\right)+\log\text{it}\left(\text{FPR}\right). \end{array}$$

The ROC is commonly used in clinical practice to evaluate the ability of a test to detect disease [30]. Until the value of this screening test is fully investigated, it is not advisable to use it as a routine test for hypertensive patients, but it is supported that a reduction in potassium is not a necessary candidate for this screening test. The flow chart of the screening test is shown in Figure 1.

First, all patients were given a detailed medical history, recording gender, age, duration of hypertension, medications taken, and treatment history. Patients were required to collect fasting venous blood at least once during hospitalization and send it to the hospital laboratory to check liver and kidney function, blood electrolytes, and blood lipids. The statistical data and clinical experience were used to determine the weights and affiliation degree affiliation function of each element in the thesis domain. Cases with weights and art weight affiliation greater than or equal to the intercept are diagnosed as PA. The basic idea is to minimize the weighted sum of squared residuals, from which the parameters are solved. Suppose that the four cells of a, b, c, and d denote TPs, FPs, FNs, and TNs, respectively, and the weights, that is, the inverse of the variance, are noted as W, and the expressions are

(5) $$\begin{array}{c} \text{W}={\left[\mathrm{var}\left(D\right)\right]}^{-1}={\left(\frac{1}{a}+\frac{1}{b}+\frac{1}{c}+\frac{1}{d}\right)}^{-1}. \end{array}$$

The estimated AUC for CCT diagnosis of PA was 0.9 and the SSST was 0.6. The sample size ratio of patients with PA to patients with essential hypertension should be 3 : 1 in subjects with an ARR ratio greater than or equal to 2.0 ng-dl^−1^/m IU-l^−1^, and the area under the curve of false positive rate between 1 and 2 was calculated. Blood was collected at 8:00 a.m. on the morning of the test day in a resting, lying, fasting state. 50 mg of Kepone tablets (Sino-US Shanghai Squibb Pharmaceutical Co., Ltd.) was taken orally after blood collection, and blood was collected again at 10:00 a.m. 2 h later to measure plasma renin activity and angiotensin and aldosterone levels. The purpose was to differentiate from adrenal malignant tumor, and then use CAH for diagnosis, as shown in Figure 2.

Secondly, all hypertensive patients were asked to discontinue all types of antihypertensive drugs for at least 2 weeks before the test, and those who could not tolerate discontinuation could be given ion channel antagonists to control blood pressure. The blood specimens for PAC and PRC should be centrifuged within 2 h of collection and tested promptly. For the blood pressure test, the subject should rest calmly for 5 minutes or more and take a seated position with one sleeve removed to expose the forearm, so that the elbow is as close to the heart as possible. The mercury sphygmomanometer was selected and placed upright to zero the reading, then the sphygmomanometer cuff was wrapped around the upper arm close to the skin so that the lower edge of the cuff was approximately 2 fingers above the transverse elbow line, and the tightness was such that 1 finger could be reached.

Finally, the patients were asked to eat and drink normally before the test, and the day before the test, the patients were asked to accurately retain hourly urine, measure urine volume, and test urine potassium and urine sodium. All subjects began fasting after 10:00 pm the night before, and blood was drawn from the elbow at 8:00 pm the next day and sent to the hospital laboratory for biochemical, lipid, glycated hemoglobin, and fasting glucose measurements on a biochemical analyzer. In hypertensive patients, the basal recumbent ratio was measured, and in patients with renin after standing (tachypnea) excitation, the diagnosis of PA was made in combination with adrenal, post-surgical pathology, and follow-up results.

### 3.2. Method of the Captopril Inhibition Test

The Kepone inhibition test is one of the most widely used clinical tests to confirm the diagnosis of proaldosteronism. It is traditionally believed that the diagnosis of primary aldehyde should include three levels of screening, confirmation, and staging, and ARR is currently the preferred method recommended by national guidelines for the first level of primary aldehyde diagnosis [31]. In the early literature of pancreatic cancer diagnosis, it was noted that PET and EUS-FNAB techniques can improve the diagnosis of PDAC, but their effectiveness is often limited by the high cost and technical difficulty. The regression parameters A and B are derived from the five equations presented above, and then the regression equation for the SROC curve can be established using the following equation:

(6) $$\begin{array}{c} \text{TPR}=\left[1+e^{-A/\left(1-B\right)}{\left(\frac{1-\text{FPR}}{\text{FPR}}\right)}^{\left(1+B\right)/\left(1-B\right)}\right]. \end{array}$$

Therefore, three confirmatory tests, SSST, CCT, and FST, were completed in the high-risk group for prodromal aldehyde, and the Kepone inhibition test was used as a reference standard to evaluate the diagnostic efficacy of SSST and CCT in the diagnosis of prodromal aldehyde and to finally determine the best diagnostic test for prodromal aldehyde. After the patients and their families gave their consent and signed the informed consent form, peripheral blood was collected from the prevalent patient, the father, and the mother for genomic DNA analysis. The genetic analysis process is shown in Figure 3.

First, gender (male/female), age (years), duration of hypertension (years), presence of hypokalemia, and medication use were recorded. Nonnormally distributed variables were expressed as medians (interquartile spacing), and the rank-sum test (*U* test) was used for comparison between groups. After fasting for at least 8 hours, patients were given 75 g of glucose powder dissolved in 250 ml of warm water orally in the early morning on an empty stomach, timed from the first sip and finished in 3–5 minutes, and blood glucose was measured on the forearm 2 hours after taking the glucose. TPR + FPR =1 was a diagonal line, and on this diagonal line, the sensitivity and specificity were equal, that is, *S*=0.

(7) $$\begin{array}{c} S=\text{logit}\left(\text{TPR}\right)+\text{logit}\left(\text{FPR}\right)=0. \end{array}$$

Namely,

(8) $$\begin{array}{c} \text{logit}\left(\text{TPR}\right)=\text{logit}\left(\text{FPR}\right). \end{array}$$

In the CTT experiment, plasma aldosterone and renin concentrations were measured in the prone position after the patient remained in the ambulatory position for at least 1 hour, and plasma aldosterone and renin concentrations were measured before the dose of 50 mg captopril at 8:00 a.m. Plasma aldosterone and plasma renin concentrations were measured again at 10:00 a.m. During the test, the patient was not allowed to lie down and eat. The standard error expression for TPR was:

(9) $$\begin{array}{c} \text{SE}\left(\text{TPR}\right)=\frac{\text{SE}\left(A\right)}{8{\left[\cosh\left(A/4\right)\right]}^{2}}. \end{array}$$

Next, blood was drawn before the test and 2 h after oral administration of 20–45 mg of captopril, and PA and PRA were measured. Logistic regression analysis was used for risk factor analysis. *p* < 0.04 was defined as a statistically significant difference, and a two-sided test was used. At this time, the accuracy of the diagnostic test could be estimated by using statistical quantities, as shown in the following equation:

(10) $$\begin{array}{c} Z=\frac{{\text{TPR}}_{1}-{\text{TPR}}_{2}}{\sqrt{{\text{SE}}^{2}}\left({\text{TPR}}_{1}\right)+{\text{SE}}^{2}\left({\text{TPR}}_{2}\right)}, \end{array}$$

where *Z* is the normal deviation value; TPR_1_ and TPR_2_ are the diagnostic accuracy indexes to be compared; and SE^2^(TPR_1_)  and SE^2^(TPR_2_) are the standard errors.

All subjects were required to complete blood biochemistry (electrolytes, liver function, renal function, etc.), plasma renin and aldosterone concentrations in the upright and prone positions, circadian rhythm of blood cortisol, 24-hour urinary cortisol and 24-hour urinary vanillyl amygdalin, saline loading or CCT, dexamethasone suppression test in some patients, and sex hormone testing. Under normal conditions, captopril inhibits angiotensin-converting enzyme, reduces angiotensin II production, and suppresses aldosterone secretion even in the presence of high renin.

Finally, blood and 24-h urine were collected from both hypertensive patients and normal controls, and blood and urine electrolytes were measured by a fully automated biochemical analyzer. Clinical case data of suspected adrenal lesions were collected and used to evaluate the sensitivity and specificity of the diagnostic model of PA data analysis, using routine postoperative pathological findings as the gold standard. After screening the case data, the investigators independently extracted relevant information (e.g., patient characteristics, relevant indicators needed for various applications or calculations, etc.) and reconstructed these data into a 2 × 2 column table using a standard format. The angiotensin-converting enzyme inhibitors, angiotensin receptor blockers, and *β* receptor blockers for more than 2 weeks and diuretics or glycopyrrolate preparations for more than 4 weeks were discontinued prior to blood collection. The true positive rate, false positive rate, true negative rate, and false negative rate were calculated by a columnar table.

## 4. Application Analysis of Data Analysis in Reliability of the PA Diagnostic Test

### 4.1. Threshold Effect Detection and Analysis

Data analysis was used to assess statistical heterogeneity between studies, and no significant heterogeneity between studies was considered when *p* ≥ 0.03. A fixed-effects model was selected for data analysis, and it was found that antihypertensive drug administration significantly affected the accuracy of the threshold effect assay. The results of two different immunological diagnostic tests, IHA and ELISA, were comprehensively evaluated using the threshold effect assay and bivariate model analysis of sensitivity and specificity in order to obtain more accurate conclusions and provide a basis for the selection of future screening methods for PA. The ROC curves of the confirmatory tests for the diagnosis of protoaldehyde and its subtypes are shown in Figure 4.

First, when using data analysis for PA screening, attention should also be paid to test method standardization and threshold setting, which varies in the literature reporting different body positions, blood collection times, etc. Threshold settings also vary. There are many ways to obtain comprehensive diagnostic test accuracy, but the more commonly used methods include comprehensive receiver operating characteristic analysis and bivariate model analysis for sensitivity and specificity. Plasma aldosterone levels do not follow a normal distribution, so they are expressed as the median of the data. Normally distributed data were expressed as mean ± standard deviation, and nonnormally distributed data were transformed for normality by taking natural logarithm values. Comparisons of plasma aldosterone levels between the proaldosterone and nonproaldosterone groups were performed by nonparametric tests. One-way ANOVA was used for comparisons between the two groups. Correlations between factors of normally distributed data were analyzed by correlation. Patients with a positive test should have an enhanced CT examination of the adrenal glands, and patients who are willing to undergo adrenalectomy are recommended to have an adrenal vein (AVS) to identify the dominant side of aldosterone secretion. Almost all patients with PA showed different degrees of hypertension, except for the early PA patients who were found to have no hypertension during the health checkup, so the difference was statistically significant, and the 2-h postprandial blood glucose level was positively correlated with the standing aldosterone level, as shown in Figure 5.

Secondly, in the case of a certain test method, the higher the threshold setting, the lower the sensitivity and the higher the specificity. Acceleration equation and acceleration factor are two very important concepts in accelerated tests, which are called accelerated life equation in accelerated life test. True classification is defined as two mutually exclusive states, such as the presence or absence of disease, benign or malignant tumor, positive or negative test results, etc. For the determination of renin activity, two copies of the same sample are taken, one at 4°C to react directly with the antibody and the other at 37°C for a period of warming before reacting with the antibody. The concentration of angiotensin I in the two samples was measured separately, and the renin activity was obtained by dividing the concentration of angiotensin I in the 37°C sample by the concentration of angiotensin I in the 4°C sample by the incubation time. The sensitivity of standing ALD and ARR for the diagnosis of PA is slightly poorer, but the specificity is better, while the sensitivity of prone ALD and ARR for the diagnosis of PA is better, but the specificity is slightly poorer (Figure 6).

Finally, other confirmatory tests must be performed after the screening test to reduce the false positive rate. The true screening status is determined by the gold standard, which is a test that is completely different from the test being evaluated and whose results are recognized by all. Patients whose true status is higher than the initial screening cut point are further tested with a confirmatory test (intravenous saline test, or CCT, or fludrocortisone suppression test). Patients with a positive confirmatory test underwent enhanced CT of the adrenal glands and, in some cases, bilateral adrenal venous blood sampling. During this period, drugs with a low effect on this ratio, such as hydrazidiazide, prazosin, and verapamil extended-release agents, could be used as needed to control hypertension symptoms. The overall sensitivity, specificity, area under the curve, and diagnostic test advantage ratio were found to be 0.87 (95% CI 0.84–0.93), 0.93 (95% CI 0.95–0.98), 0.94, and 371.13, respectively, but heterogeneity was evident.

### 4.2. Statistical Analysis of Diagnostic Reliability

The purpose of diagnostic tests is to explore easy, quick, and cost-effective methods for early diagnosis, but their diagnostic value can be influenced by various factors, such as disease spectrum, gold standard, and outcome evaluators. The results of different studies suggest that the diagnostic efficacy of ADRR in PA screening is highly variable; there is also controversy over the need to discontinue medication in patients taking hypotensive drugs when measuring ADRR values. The clinical threshold for screening is generally set at 30, and a diagnosis of prodromalgia is confirmed if the patient's ARR is greater than 50. Therefore, it is necessary to analyze the data on the diagnostic efficacy of ADRR in PA to clarify the role of ADRR in proaldosterone screening. The septal thickness and left ventricular weight index of PA patients were higher than those of EH patients, with statistically significant differences, and there was a positive correlation between standing and lying ALD levels and septal thickness (see Figure 7).

First, threshold effects were assessed using Spearman's correlation coefficient, using *I*^2^ values to assess heterogeneity between included studies ranging from 0% to 90%, with 0% indicating no heterogeneity and more than 40% indicating significant heterogeneity of included studies. Renin and aldosterone levels were influenced by a variety of conditions that were not uniformly controlled for in the study, including the use of antihypertensive medications, blood sample collection from outpatients or inpatients, timing of blood collection, body position during the trial, sodium and potassium intake, and menstrual cycle. Any new diagnostic technique or new diagnostic method formally applied in clinical practice needs to be evaluated for methodological quality and clinical applicability using scientific, standardized, and rigorous methods. A random-effects model was used when significant heterogeneity between studies was considered at *p* < 0.06. Deek's funnel plot was used for diagnostic tests to determine whether there was significant publication bias. Diagnostic accuracy was improved, thus guiding physicians to take correct and reasonable decisions for patients during clinical treatment. Patients had higher SUSPUP as well as SUSPPUP compared with patients with primary hypertension, with statistically significant differences, and the ROC curves of each index in PA screening are shown in Figure 8.

Second, the efficacy of PA screening for ADRR was assessed using the combined total sensitivity and total specificity, expressed as an 85% confidence interval. A dramatic increase in fluid volume can suppress blood aldosterone secretion to a large extent, while antihypertensive drugs have little effect on the results of this test. The design of the diagnostic test is unique, and its internal and external validity is susceptible to numerous factors.

The aldosterone levels were significantly higher in PA patients than in patients with essential hypertension, and the differences in blood and urine electrolytes were statistically significant. The blood potassium levels were lower in PA patients than in those with essential hypertension, while the blood sodium, urine sodium, and urine potassium levels were higher in PA patients than in those with essential hypertension. The comparison of the area under the curve of each index as well as the optimal cut point and sensitivity and specificity of each index are shown in Tables 1 and 2.

The diagnostic advantage ratio is the ratio of the positive likelihood ratio to the negative likelihood ratio and is the best indicator to evaluate the efficacy of a diagnostic test. In studies containing multiple PA subtypes, a higher APA ratio will result in a higher specificity and a lower sensitivity of the diagnostic cut point. Flawed trial design, inappropriate subject selection, poor trial execution, inappropriate data analysis, and poor interpretation of study results may lead to misestimation of trial accuracy, resulting in premature application of immature diagnostic tests to clinical practice with harmful clinical consequences.

Finally, forest plots were used to indicate the sensitivity and specificity of all included studies. The mechanism could be the low level of aldosterone secretion and the weak autocrine capacity in patients with normal blood potassium. When post-saline PAC and post-cato PAC were used to confirm the diagnosis of prodromal, respectively, there was a similar area under the subject working curve between SSST and CCT, 0.89 and 0.78, respectively, with no significant difference in the area under the curve between the two (*p*=0.546). Data analysis was used in the significant variable regression analysis to establish the scoring system predicting prodromal. The row variables of the column table reflect the true classification status of the patients, that is, the gold standard test results; while the column variables are the diagnostic results of the evaluated tests, noted as positive versus negative.

## 5. Conclusions

With the intensive study of PA, it is now believed that PA is a common cause of secondary hypertension, and its prevalence is about 6%–15% of hypertensive patients. Compared with typical UPA patients, patients with CT-negative unilateral PA have milder clinical symptoms, and an increased number of APCC is an important pathological feature. The diagnosis of PA is a complex process, especially in patients with mild clinical symptoms and no hypokalemia, and the diagnosis needs to be made by combining the results of multiple tests and comprehensive analysis to guide treatment. Therefore, this study proposes a data analysis-based reliability analysis of functional diagnostic tests for PA, incorporating proaldosterone cases, using data analysis to obtain eigenfunction coefficients, exploring new methods for proaldosterone screening and diagnosis, and conducting an in-depth study on the diagnostic reliability of medical mathematization. The combined use of data analysis would improve the reliability of test results, and data analysis-based reliability analysis of PA functional diagnostic tests is a more feasible option because it is safer and easier to implement. In conclusion, this study is a guideline for the screening of PA and provides a viable basis for the clinical development of plasma renin concentration screening for the disease.

## Figures and Tables

**Figure 1:** Research flow chart.

**Figure 2:** CAH diagnosis flow chart.

**Figure 3:** Gene analysis process.

**Figure 4:** ROC curve of a diagnostic test for protoaldehyde and its subtypes.

**Figure 5:** The correlation between blood glucose at 2 h after meal and ALD in upright and supine positions.

**Figure 6:** ROC curve of diagnostic PA drawn by ALD and ARR values in upright and supine positions.

**Figure 7:** Comparison of ventricular septal thickness between PA and EH.

**Figure 8:** ROC curve of each index in PA screening.

**Table 1:** Comparison of the area under the curve of each index.

Index	ARR	Blood sodium/potassium	SUSPUP	SUSPPUP
AUC	0.876	0.782	0.694	0.578
SE	0.03	0.02	0.02	0.04
*p* value	<0.01	<0.01	<0.01	<0.01

**Table 2:** The best cutoff point, sensitivity, and specificity of each index.

	ARR	SP	SPP
Optimum tangent point	29.68	46.26	15.36
Sensibility	1.04	0.87	0.68
Specificity	0.897	0.765	0.695

## Data Availability

The dataset can be accessed upon request.
